RETRACTED

# The Construction of Ecosystem and Collaboration Platform for Enterprise Open Innovation

**DOI:** 10.3389/fpsyg.2022.935644

**Published:** 2022-07-07

**Authors:** Maoxiang Wang, Ruili Zhang, Rasheed Abdulwase, Shuangsheng Yan, Mohsin Muhammad

**Affiliations:** ^1^School of Economics and Management, Southeast University, Nanjing, China; ^2^China Mobile Group Jiangsu Co., Ltd., Nanjing, China; ^3^School of Health and Economics Management, Nanjing University of Chinese Medicine, Nanjing, China; ^4^School of Management, Jiangsu University, Zhenjiang, China; ^5^Marxism School, China Pharmaceutical University, Nanjing, China; ^6^Business School, China Pharmaceutical University, Nanjing, China; ^7^School of Finance and Economics, Jiangsu University, Zhenjiang, China

**Keywords:** open innovation, ecosystem, collaboration platform, user-collaborative innovation, commercialization

## Abstract

In the era of the knowledge economy that is filled with intense competition, formal closed innovation can no longer meet the market demand. The enterprise needs to implement open innovation involving external resources. The concept of open innovation emphasizes both the use of internal and external resources in the process of enterprise innovation and the use of internal and external markets to promote the commercial application of innovation achievements. With the rapid development of Internet technology, enterprises must build an open innovation ecosystem of benefits-sharing, identify, connect, and utilize external innovation resources, and be committed to creating an open innovation ecosystem without organizational boundaries. Enterprises should pay attention to coordinating the relationships among the innovation ecosystem members, eliminating heterogeneous barriers between enterprises and their partners, and enhancing their cooperative innovation ability with external organizations. It is also necessary to build a collaborative innovation platform convenient for the release and acquisition of innovation information, the collection of customer needs and related ideas, and the full use of external resources for innovation. In particular, it is necessary to guide users and related resources to the innovation platform, realize the maximum effect of resource aggregation, and promote customer demand-oriented new product development. Through building an open innovation ecosystem and a collaboration platform, it is helpful for enterprises to seek all kinds of technical and resource support, enhance their ability of independent innovation, promote the emergence of many innovative achievements, and realize value co-creation and win-win cooperation with partners.

## Introduction

In the era of fierce competition in the knowledge economy, enterprises cannot meet the market demand only by relying on the traditional closed innovation. They need more and more external resources to participate in innovation. By implementing open innovation, acquiring externally differentiated knowledge, and seeking collaborative innovation with external organizations, enterprises will be able to quickly respond to market demand and maximize commercial profits. The first proposed the concept of “open innovation” from the enterprise level and defined it as “the purposeful inflow and outflow of knowledge to promote internal innovation and expand the external application market of innovation.” Çubukcu et al. (2021) believed that open innovation emphasizes the connection and integration of multidisciplinary knowledge inside and outside the organization. The more forthcoming the innovation process is the more information, knowledge, technology, and innovation-related intangible assets the enterprise obtains from the external organization, which will improve the enterprise’s innovation performance. Gusmeroli (2012) pointed out that open innovation broadens the ways, opportunities, and capabilities of the organization’s policy-making, increasing the innovation revenue significantly. As early as the beginning of this century, many enterprises in European and American countries began to study and practice open innovation modes and have achieved commercial success. The success of globally excellent innovative enterprises, such as P&G, 3M, and Intel, is all related to the open innovation strategy with openness, cooperation, and sharing.

RETRACTED

Denhere (2016) pointed out that the development tendency of technological innovation in the twenty-first century is open innovation. The continuous development of the Internet and other emerging technologies provides favorable conditions for enterprises to realize open innovation. pointed out that open innovation will bring a series of thinking reforms and social issues. Through the analysis of multiple cases, Risfandhani (2016) found that enterprises must successfully implement open innovation and build a network system of the collaborative invention and an ecosystem of open innovation. Balla (2016) pointed out that all kinds of innovation elements, namely, knowledge, skills, and resources, are separated in space and organization, and enterprises should build a strong innovation network to integrate and apply them. At the same time, enterprises must build a collaboration platform to promote the opening-up and sharing of resources between enterprises and relevant partners. In this way, enterprises can facilitate the effective accumulation of innovation elements in all aspects, effectively integrate with external innovation resources, encourage customers to participate in innovation activities effectively, and improve innovation effectiveness in a better way.

RETRACTED

## The Connotation and Characteristics of Open Innovation

The concept of open innovation emphasizes the use of internal and external resources in the process of enterprise innovation and the use of internal and external markets to promote the commercial application of innovation results. Considering the wide distribution of innovation resources, it is difficult for any organization to play the role of innovation alone. Organizations must cooperate and open their internal innovation resources to each other. The process of open innovation is the process of integrating the internal and external resources of the enterprise. In this process, enterprises should strengthen internal and external collaborative innovation and extensively use the internal and external technology, creative ideas, and resources (Hilbers et al., 2019; Khosravi et al., 2019; Kordej-De Villa and Slijepcevic, 2019; Ozoike-Dennis et al., 2019).

Analyzing from the knowledge perspective, Rahmah (2018) described open innovation as a knowledge management activity of “knowledge exploration → knowledge retention → knowledge application.” Wawan (2016) believed that open innovation is a multi-agent innovation based on innovation cooperators, and more innovation elements should be absorbed. Leonidou et al. (2020) believed that open innovation can promote enterprises to become more integrated with the external knowledge networks. Melendez et al. (2019) pointed out that in open innovation, enterprises should pay attention to the information of their resources to obtain more benefits from external cooperation. Solaimani et al. (2019) believed that open innovation means that enterprises systematically collect and integrate relevant customer information to generate ideas. Based on the industry type and enterprise scale analysis, Appio et al. (2021) believed that open innovation includes industry university research cooperation, strategic alliance, R&D outsourcing, supplier participation, enterprise merger and acquisition, and other modes. They believed that open innovation is the flow and integration of innovation resources between enterprises and their innovation partners (Mohsin et al., 2020, 2021).

Believed that open innovation can be deconstructed into openness, cooperation, and innovation. Openness is reflected in breaking through the boundaries of enterprises, including the openness of the innovation environment, resources, subjects, and creative ideas (Mohsin et al., 2022a,b). “Openness” is a variable that characterizes the degree of openness in the process of open innovation, which includes two dimensions, namely, “depth” (the degree of openness in a particular field) and “breadth” (the category of open fields). Keupp and Gassmann took the difference in open innovation’s breadth and depth as the classification benchmark. They identified four types of open innovation (Figure 1), namely, isolators (low breadth and depth of open innovation), scouts (low depth and medium high breadth), explorers (medium depth and medium high breadth), and professional innovators (high breadth and depth) (Nambisan et al., 2017; Sun et al., 2019; Tiep et al., 2021) pointed out that the higher the openness of enterprises, the more cooperation with partners in different industries or regions enterprises can reach. Johannsen et al. (2021) pointed out that open innovation requires innovation subjects to be open and requires innovation subjects to actively cooperate with partners from an open perspective.

RETRACTED

**FIGURE 1:** Keupp and Gassmann’s classification of open innovation types (Keupp and Gassmann, 2009).

The concept of open innovation is relatively general. Any non-closed innovation activities of enterprises can be regarded as open innovation, such as joint research and development, acquisition or output of intellectual property rights, and acquisition of new ideas or even new products, allowing third parties to develop software or services. In terms of basic principles, Table 1 shows the differences between closed innovation and open innovation (Sitthisomjin et al., 2020). Through the implementation of open innovation, enterprises’ external complementary resources and advantageous internal resources are put in the same important position so that enterprises can save innovation costs and improve innovation efficiency (Baloch et al., 2020; Sun L. et al., 2020). Enterprises can focus on their strengths and “comparative advantage” areas for innovation, reducing the risk of innovation and improving the chance of innovation success.

**TABLE 1:** The comparison of the basic principles of open innovation and closed innovation.

Basic principles	Closed innovation	Open innovation
Corporate philosophy	Develop good products by oneself, etc.	The best ideas may come from elsewhere.
Innovation resources	Pay attention to the enterprise’s internal resources and do research by one’s own.	Integrate global resources to innovate.
Core competence	Vertical integration of product and service design.	The ability to search, identify, acquire, and utilize external resources; integrating internal and external resources.
Responsibilities of employees	Complete the top-down tasks.	The subject of enterprise innovation.
Roles of users	Passively accept the products of enterprises.	Take the initiative to carry out collaborative innovation with enterprises.
Measurement of innovation success	Increased revenue or profits; Reduced time to enter the market; Market share.	Return on R&D investment; Break-through innovative products or business models.
Intellectual property rights	Own and strictly control intellectual property rights.	Buy ‘others’ intellectual property and make profits by selling the intellectual property of one’s own.

With the continuous development of information and network technology, the collaborative innovation relationship between enterprises and external organizations has become closer, and an innovation ecosystem with symbiotic relationships breaking through the traditional regional, industrial, and national restrictions is forming gradually (Alemzero et al., 2020; Sun H. et al., 2020). Enterprises should gather their upstream and downstream external resources to build an open and innovative ecosystem; realize networked collaboration among organizations within the system; and realize the effective integration of human resources, technology, information, capital, and other creative elements (Agyekum et al., 2021; Zhang et al., 2021). In addition, with the increasing of technological complexity and market dynamics, the interaction of the leading bodies in the innovation ecosystem is increasingly frequent and in-depth, the scope of innovation subjects in the innovation ecosystem is more comprehensive, and the flow of innovation resources is more frequent (Chien et al., 2021; Iqbal et al., 2021; Li et al., 2021). The operation of the innovation chain is more complex. It is necessary to build a collaborative innovation platform to realize the effective convergence of innovation factors on the platform to achieve better cooperation for open innovation (Chandio et al., 2020; Sun H. et al., 2020).

RETRACTED

## The Path of Constructing an Open Innovation Ecosystem

### Clarify the Primary Connotation of the Open Innovation Ecosystem

Defines an ecosystem as a system in which companies are symbiosis, and they meet customer’s needs and obtain economic value through the interaction between individuals and others. Pointed out that in the process of open innovation, enterprises should be committed to creating an open innovation ecosystem without “organizational boundaries.” Jacko (2020) pointed out that the open innovation ecosystem includes the business ecosystem and R&D ecosystem. Enterprises should focus on building an open innovation ecosystem in the existing business ecology and expand innovation effectiveness with joint ecosystem efforts. With the rapid development of Internet technology, it is necessary to understand the dynamic evolution process of the innovation ecosystem from the perspectives of technological change and the social division of labor. The Internet has made it easier to deliver ideas and deploy global resources, making large-scale open, collaborative innovation (Iqbal et al., 2021; Zhang et al., 2021).

By building an open innovation ecosystem with collaborative cooperation, resource optimization, benefit-sharing, and win-win, more highly specialized individuals can focus on more refined fields to participate in innovation, and enterprises can achieve value creation effects that a single organization cannot reach. Therefore, enterprises should pay attention to the identification, connection, and utilization of external innovation resources as part of the innovation ecosystem to enhance the innovation speed and intensity of the whole system (Ehsanullah et al., 2021; Hsu et al., 2021; Zhang et al., 2021). For example, IBM has been integrating global innovation resources since 2003, expanding innovation activities beyond the scope of the company and building IBM’s innovation ecosystem (Figure 2), which has successfully promoted the transformation of enterprises from hardware vendors to solution providers. In the process of open innovation, enterprises should especially pay attention to inviting customers to participate directly, truly understanding the customer’ needs and further clarifying the direction of innovation.

**FIGURE 2:** IBM’s innovation ecosystem (IBM Annual Report).

### Coordinate the Relationship Between the Enterprise and Its Partners

Enterprises play an irreplaceable role in the open innovation ecosystem and are the main participants in knowledge innovation, diffusion, and application. Enterprises have the leading power in selecting partners, task allocation, and benefit allocation in the ecosystem. Partners refer to the participants in the innovation network, usually as the subsidiary roles of enterprises in the innovation ecosystem. Open innovation provides more innovation development opportunities for some partners who lack knowledge and provides support for the improvement of their innovation ability. Of course, many partners are turning from the receiver of knowledge spillover to the exporter of knowledge spillover, which is more and more common.

Government departments should play their leading and coordinating roles, promote the improvement of the internal structure of the open innovation ecosystem, promote the efficient integration of complementary knowledge between enterprises and their partners, and promote the construction of a scientific, practical, and standardized distribution mechanism of innovation benefits. Government departments should formulate related policies to support enterprises and partners to carry out forward-looking and leading innovation and guide them to pay attention to the commercial transformation of innovative achievements. At the same time, enterprises should build a compensation mechanism to accelerate the convergence of partners and innovation elements into the innovation ecosystem.

RETRACTED

### Eliminate the Heterogeneous Barriers Between Enterprise and Its Partners

In the open innovation ecosystem, the heterogeneity of partners (including the heterogeneity of industries) will impact innovation effectiveness. Partners’ unique and different knowledge can promote complementary advantages, resource sharing, and win-win cooperation among heterogeneous organizations and bring greater benefit space to collaborative innovation. However, when enterprises carry out collaborative innovation with more and more heterogeneous external organizations, they may have an “exclusive” response to heterogeneous knowledge resources. It is difficult for heterogeneous knowledge resources to connect with the existing knowledge systems of enterprises, which is not conducive to the improvement of open innovation performance, so it should be resolved.

With the continuous advancement of open innovation, enterprises should constantly accumulate cooperation experience with heterogeneous partners and optimize their cooperation mode. In the innovation ecosystem of industry-university research cooperation, universities and scientific research institutes have strong scientific research abilities, which are heterogeneous compared to enterprises. Enterprises should pay attention to eliminating heterogeneity and improving their cooperative innovation ability. In open innovation, enterprises should also cultivate organizational learning abilities and enhance the ability to identify, integrate, and share all kinds of information, which will help enterprises eliminate all types of heterogeneous barriers, fully absorb and digest external knowledge, and integrate the external expertise into the existing resource structure to maximize the benefits of collaborative innovation.

### Promote Cooperative Innovation of Internal and External Talents

In the open innovation ecosystem, enterprises should fully absorb external innovation resources and talents, vigorously introduce high-end international skills, and improve the utilization efficiency of human resources. At the same time, enterprises should strengthen the cultivation of innovative talents, promote the cooperation of internal and external skills to carry out innovation, and constantly stimulate the innovation vitality of talents (Wasono and Furinto, 2018). It is necessary to promote the innovation behavior of innovative talents from the past passive interest driven to the internal drive of self-value realization to achieve a win-win situation between enterprises and creative talents.

RETRACTED

For example, Haier’s innovation can be carried out by employees inside the enterprise or by talents worldwide, and Haier can fully use external talents. Haier’s open innovation subverts the traditional closed concept of talents and reflects the cross-border integration of talents. Haier attracts countless talents from all over the world to develop in Haier every year, and Haier has become a global gathering place for innovative talents. Haier realizes the dynamic match between talent supply and market demand by building a dynamic talent circulation system that adapts to the real-time dynamic characteristics of self-organization and self-circulation of open innovation. According to the needs of market development and personal value realization, internal staff in Haier will actively participate in innovation activities.

### Enhance the Cooperative Capabilities of Enterprises and External Organizations

In the open innovation ecosystem, enterprises must pay attention to improving the ability of collaborative innovation to ensure gaining competitive advantage more quickly in innovation. The stronger the enterprise’s innovation ability is, the easier it is to introduce external innovation resources in the open innovation process. The stronger the attraction of collaborative innovation to external institutions. Zhou et al. (2021) believed that under the conditions of open innovation, innovation capabilities can be divided into absorption capability, conversion capability, and diffusion capability. First proposed absorption capability and defined it as the ability of an enterprise to search, absorb, and commercialize external knowledge. Rose et al. (2020) pointed out that absorption capability refers to the dynamic ability of enterprises to identify and utilize external technological opportunities. Conversion capability refers to enterprises’ ability to redefine product technology based on internal options continuously. Diffusion ability refers to the power of innovation results to spread in a potential user group through a certain way of communication. Innovative achievements can be better commercialized through the external application of new knowledge, new technology, and new products.

The successful practice of many companies shows that enhancing absorptive capacity is extremely important for the construction of open innovation. Frishammar et al. (2019) divided absorptive capacity into five processes: identification, acquisition, absorption, transformation, and utilization of knowledge and resources. When an enterprise has a deep knowledge base in a particular field, it shows that, in this field, the enterprise has a good understanding and use of this knowledge and has a strong ability to absorb and understand the new knowledge in this field. By strengthening knowledge acquisition, knowledge learning, and knowledge sharing, it is helpful for enterprises to transform external knowledge into internal knowledge to achieve a pleasing effect of knowledge innovation.

RETRACTED

## Architecture and Applications of Innovation Collaboration Platform

### Architecture Characteristics of Innovation Collaboration Platform

Melendez et al. (2019) pointed out that the “platform” is an aggregation of “soft” and “hard” elements. An enterprise needs to build a collaborative platform to provide a virtual environment for open innovation. Innovators can express their suggestions and relative ideas to improve products and services in the forum. The platform innovation mode has changed the original one-way innovation mode to a parallel R&D model, which focuses on gathering users and resources for the platform and letting them deeply participate in the product development. Building a collaborative innovation platform based on openness, cooperation, innovation, and sharing can promote the mutual attraction and matching of various innovation resources and encourage enterprises to effectively collect market demand and innovation programs. Enterprises in the core position of the platform can enjoy more resources and information, effectively connect and restructure them, and quickly launch new products to meet the needs of users with the help of external forces.

### Comprehensive Application of Innovation Collaboration Platform

At present, many enterprises attach great importance to building their innovation platform and promoting the platform’s collaborative application. For example, Appio et al. (2021) has created a new generation of AI innovation platforms, created an open system of product operating and an available algorithm ecological environment, helped zero algorithm primary users develop their intelligent industry algorithms, and helped AI practitioners and entrepreneurs have their smart hardware products and solutions. Cisco selects a hosting platform for creative idea management for Bright Idea Company to let customers express their ideas, participate in product design, plan marketing activities, and jointly develop products on the platform. Lego has also established a “design by me” platform. Customers can download the software from the platform, upload their ideas to the forum, and integrate their ideas into Lego’s new product. P&G innovatively builds a “contact and development” platform, advocates the transformation of R&D mode into C&D (connect + develop) mode, and realizes the platform’s internal and external collaborative innovation.

RETRACTED

Haier has built a typical collaborative innovation platform and formed a Haier open partnership ecosystem (HOPE) earlier in China. In the forum, one end is connected with the potential needs of different users globally, and the other is associated with the world’s top R&D personnel and resources. The technology demander and the technology provider are precisely matched. Solaimani et al. (2019) analyzed the design idea of HOPE based on modularization under the background of the network. HOPE is divided into modules of community interaction, technology matching, and creative idea transformation, which makes it convenient to capture the latest technology trends, realize the sharing and connection of innovation knowledge, and realize the rapid matching of innovation resources (Figure 3). The interaction module of the platform represents the platform gathering a large number of users and external institutions to participate in various interactive activities. Through the analysis and collation of the background data, enterprises can fully understand the needs of multiple users and then carry out product planning. The technology matching module contains the technology resources and the corresponding technical solutions registered on the platform. Through the big data matching analysis, any user demand can be quickly and accurately compared to the appropriate solution after being sent to the platform. The creative idea transformation module means integrating user demand information and technical solution information on the platform, putting forward feasible product solutions, and quickly developing the required new products.

**FIGURE 3:** Module composition of HOPE.

### User Collaborative Innovation Based on Platform

Put forward the concept of user innovation in 1994. They thought enterprises should pay special attention to letting users participate in product design, innovation, and R&D. The integration of creative ideas of enterprises and customers is particularly important to ensure better that the innovation of products is close to the needs of users. The cooperation between enterprises and customers can promote more innovative achievements with rich connotations and high complexity. Public customers can use the collaboration platform to publish the relative ideas and carry out highly interactive and cooperative innovation with enterprises. Technical personnel scattered in different geographical locations around the world gather in the collaboration platform to engage in research work in their areas of interest, form a development community of professional knowledge, and promote customer demand-oriented development of new products, which can help enterprises achieve the goal of rapidly occupying the market (Scafuto et al., 2020).

RETRACTED

For example, Lego is a family-owned private enterprise in Denmark. It is a global leader in providing high-quality products and experiences that stimulate children’s creativity, imagination, and learning ability. With the help of the collaborative innovation platform, the company often invites customers to suggest improvements to the products. Another example is that Xiaomi, as a typical domestic smartphone production enterprise, attaches great importance to the concept of “let users participate and let users cool.” By building an innovative, collaborative platform and allowing users to participate in innovation on the forum, its smartphones can adapt to users’ diverse and changing needs. Xiaomi deeply understands that using the traditional innovation model cannot meet users’ diversified requirements in the face of such a huge group as hundreds of millions of users. By constantly strengthening communication with customers and allowing customers to participate in innovation, the products better meet customers’ needs.

## Conclusion

Open innovation has become a new paradigm of enterprise innovation. Compared with the previously closed invention, its innovative resources, technology, and talents can appear worldwide. Its mode shows real-time dynamic characteristics, which dramatically improves the innovation effectiveness of enterprises. At present, the technology R&D networking and decentralization trend require an enterprise to break its boundaries and implement open innovation. The transformation of closed innovation to open innovation is the fundamental transformation of enterprise strategy. By building an open innovation ecosystem and strengthening the organizations’ cooperation, the enterprise can promote the rational flow of innovation resources and realize multi-agent collaborative innovation. Open innovation can facilitate effective collaboration between enterprises and external resources, information communication, and resource sharing, help enterprises absorb more innovative elements, and enhance the ability of independent innovation.

With the rapid development of Internet technology, enterprises should pay attention to the construction of an open innovation ecosystem, strengthen the contact with external organizations, fully absorb and utilize superficial knowledge, and develop products with the help of external forces, especially the collaborative innovation of users to ensure the best user experience of products. At the same time, enterprises should pay attention to building a collaborative innovation platform and using the platform to release and obtain innovation information, solicit customer needs and related ideas, and seek technical and resource support. The platform can enable global users and resources to achieve zero-distance interaction, achieve the maximum effect of resource aggregation, promote many innovation achievements, and realize the value of co-creation and win-win cooperation between enterprises and partners (including customers).

RETRACTED

## Data Availability Statement

The original contributions presented in this study are included in the article/supplementary material, further inquiries can be directed to the corresponding author.

## Author Contributions

SY: conceptualization, investigation, resources, writing—review and editing, and supervision. SY, MW, and RZ: methodology. MW and RZ: formal analysis. RZ: project administration. All authors have read and agreed to the published version of the manuscript.

## Conflict of Interest

MW was employed by the China Mobile Group Jiangsu Co., Ltd. The remaining authors declare that the research was conducted in the absence of any commercial or financial relationships that could be construed as a potential conflict of interest.

## Publisher’s Note

All claims expressed in this article are solely those of the authors and do not necessarily represent those of their affiliated organizations, or those of the publisher, the editors and the reviewers. Any product that may be evaluated in this article, or claim that may be made by its manufacturer, is not guaranteed or endorsed by the publisher.
